# Therapeutic potential of microalgae-derived natural compounds in diabetic wound healing: A comprehensive review

**DOI:** 10.1016/j.heliyon.2025.e42723

**Published:** 2025-02-14

**Authors:** Jinjin Pei, Simab Kanwal, Ramachandran Sivaramakrishnan, Kasinee Katelakha

**Affiliations:** a Qinba State Key Laboratory of Biological Resources and Ecological Environment, 2011 QinLing-Bashan Mountains Bioresources Comprehensive Development C. I. C., Shaanxi Province Key Laboratory of Bio-Resources, College of Bioscience and Bioengineering, Shaanxi University of Technology, Hanzhong, 723001, China; b Institute of Nutrition, Mahidol University, Salaya, Phutthamonthon, Nakhon Pathom, 73170, Thailand; c Laboratory of Cyanobacterial Biotechnology, Department of Biochemistry, Faculty of Science, Chulalongkorn University, Bangkok, 10330, Thailand; d Centre for Global Health Research, Saveetha Medical College and Hospital, Saveetha Institute of Medical and Technical Sciences (SIMATS), Saveetha University, Chennai, Tamil Nadu, India; e The Halal Science Center, Chulalongkorn University, Bangkok, 10330, Thailand

**Keywords:** Microalgae, Diabetic wound healing, Bioactive compounds, Hydrogels, Wound care

## Abstract

A variety of cell types and chemical systems are known to interact throughout the complex process of wound healing. In addition to being very uncomfortable for patients, wounds that do not heal properly or become chronic can place a heavy burden on society. The creation of novel treatment approaches can expedite the healing process, reduce the societal burden, and improve patient outcomes. Due to advancements in the field of biomedical science, microalgae have significant potential for use in diabetic wound healing and other wound healing applications. This review delves into the physiological process of wound healing, the use of microalgae in wound healing, and a detailed explanation of the wound healing roles of various microalgal originated bioactive compounds including alginate, pigments, fatty acids, proteins, polysaccharides, flavonoids and phenols. The study discusses the efficacy of photosynthetic hydrogels in drugs and oxygen delivery to the wounded area that is crucial for promoting a good healing process, as well as highlights the drawbacks and challenges involved in using microalgae for wound healing. Given the current state of the art in utilizing microalgae for wound care, this review provides new perspectives for further research, along with insightful advice and innovative suggestions for academics engaged in this area.

## 1 Introduction

Photosynthetic organisms that range in length from several to hundreds of microns are known as microalgae. Microalgae are extremely adaptable and widely distributed, making them present in nearly every kind of environment. Numerous sectors, including biomedicine, food, cosmetics, pharmaceuticals, and nutraceuticals, have found broad uses of microalgae. This is mostly due to the beneficial biological characteristics of particular microalgal species, such as photosynthesis, high biocompatibility, an active surface, and bioactive substances like proteins, fatty acids, vitamins, and other secondary metabolites [1,2].

Microalgal bioactive compounds have generated a great deal of interest due to their numerous potential medical applications. Microalgae serve as source of a diverse range of bioactive chemicals, including carotenoids, polyunsaturated fatty acids (PUFAs), polysaccharides, phenolics, and vitamins. The anti-inflammatory, antioxidant, anti-tumor, anti-viral, and radioprotective properties of these substances have been associated with potential therapeutic uses [3].

Injuries can result in bleeding, infection, scarring, and a prolonged period of time for the injured tissues to recover and regenerate, and also represent the primary clinical problems associated with morbidity [4]. Tissue remodeling, proliferation, inflammation, and hemostasis are the four stages that make up the intricate wound-healing procedure. Moreover, cells, mediators, cytokines, and growth factors are needed [5,6]. Wound dressings are crucial for promoting a good healing process to address the growing problem of wounds. A moist environment promotes the rapid wound healing processes of angiogenesis, collagen formation, and prevents dehydration [7,8]. In case of a diabetic chronic wound, owing to high blood glucose levels and an imbalance in the body redox system, excessive reactive oxygen species (ROS) are produced that result in severity of local infection and neurotoxicity [9]. Diabetes-related wounds may cease healing at any time during the normal healing phases and exhibit indications of a prolonged inflammatory response. In this scenario, various microalgal derived bioactive compounds and materials are found useful to counteract such factors that impede healing. Such as photosynthetic microalgal hydrogels, that are solid frameworks and can be either biodegradable or non-biodegradable. They are highly biocompatible and provide a tangible platform for the immobilization and adsorption of biomolecules such as growth factors, proteins, and other physiologically active biomaterials [10,11]. Because of their special three-dimensional (3D) porous matrix, flexibility, and high water content, hydrogels can mimic human soft tissues. For this reason, studies have been conducted to determine if they could be useful materials for wound healing and the delivery of specific drug applications [12]. One of the challenges in wound healing is preventing infections; antimicrobial wound dressings can aid in this area. This review discusses the biological applications of various stimulus-responsive microalgae bioactive chemicals and their potential for diabetic wound healing. The components that contribute to diabetic wound healing, a brief overview of the preparation procedures of various bioactive compounds, and an emphasis on the use of diverse stimulus-responsive microalgal bioactive compounds is also discussed here.

## 2 Healing mechanisms

### 2.1 Normal wound healing

Wound healing is a complex and dynamic physiological process that involves interactions between various cell types, growth factors, chemokines, and extracellular matrix components (ECM). Hemostasis, inflammation, proliferation, and remodeling are the four sequential and overlapping phases in the healing process of a typical wound, as described in a previous study [13]. During the bleeding stage of a wound, platelets clump together and adhere to the damaged blood vessels. This causes the blood vessels to release a variety of chemicals, including coagulation factors from exudate, which coagulate at the site of the wound and initiate a coagulation cascade reaction. When coagulation fibrin is formed from coagulation cascade components, keratinocytes and other cells migrate to the wound surface to serve as a temporary scaffold. These cells store the growth factors that they secrete, which stop the bleeding and temporarily shield the wounded region [14].

Two types of inflammatory cells that proliferate into macrophages during the inflammatory phase are neutrophils and monocytes, which are drawn to the wound (Fig. 1) [15]. These macrophages release proteases that are lethal to bacteria, injured endogenous tissues, and wound debris. They also emit ROS, which have antibacterial properties. Furthermore, they generate growth factors and cytokines that facilitate cell migration and tissue proliferation, paving the way for the development of angiogenesis and tissue granulations. Fibroblasts and keratinocytes produce granulation tissue, which resembles buds, on the wound surface during the wound proliferation phase to replace lost or injured tissue. Until they reach the wound surface, the basal cells inside and surrounding the wound will keep growing and migrating, eventually giving rise to epithelial cells [16]. Furthermore, the rates of collagen deposition, degradation, and microvascular or capillary expansion are lower in the area around the wound than the rate of collagen formation, mostly of collagen III. Collagen's composition shifts from type III to type I throughout the remodeling phase [17]. Because type I collagen has a higher tensile strength, scars near the site of injury eventually fade due to the increased tensile strength in that area. During this time, the blood vessels and related cellular populations gradually diminish as the skin slowly recovers to its normal state.

**Fig. 1:** Comparison between various stages of healing in normal and diabetic wounds. Adapted with permission from Ref. [15].

### 2.2 Diabetic wound healing

ROS are produced excessively by the body due to an imbalance in the redox system and high blood glucose levels. Consequently, a high oxidation environment develops in diabetic chronic wounds, leading to local infection, vascular dysfunction, and neurotoxicity, all of which impede the healing process [9]. Following an injury, the initial stages of skin healing include hemostasis and inflammation. Aggregated platelets release a platelet-derived, transforming and epidermal growth factors as well as proinflammatory cytokines. These substances draw inflammatory cells to the wound site, where they mature into macrophages, which destroy infections, foreign objects, and injured endogenous tissues. These cells include neutrophils and monocytes [18]. Moreover, fibroblast, platelet-derived and transforming growth factor are released by neutrophils and macrophages which helps in wound healing [19]. Neutrophils are stimulated during ECM leaching by chemotactic signals. With the help of cell adhesion molecules, they then roll and migrate around the perimeter of the circulatory system, filling the wound site and producing adhesion in the process. But in diabetics, the decreased circulation at the site of the lesion prevents neutrophil adherence, leading to protracted inflammatory phases that further impede the healing cascade as illustrated in Fig. 1 [15].

Local growth factor signals drive fibroblasts and keratinocytes to the wound surface, where they multiply, release collagen fibers and ECM, and form granulation tissue adjacent to newly formed blood vessels [20]. A study discussed *ex vivo* and *in vitro* models of murine diabetic tissue wound healing and their impact on cellular calcium signals through live cell imaging. When compared to non-diabetic controls, diabetic cells showed a decrease in calcium signaling propagation. Further investigation showed that the purinergic receptor P2X7 expression in diabetic cells is responsible for wound healing. This alteration of expression and calcium signaling can explain the diabetic wound response aberrations [21].

## 3 Physiology of diabetic wound healing

The human skin, which has the largest surface area of any organ, is essential for shielding the internal organs [22]. As the body's first line of defense, the skin is particularly vulnerable to damage from Ultraviolet (UV) radiation, microbial infections, and mechanical stress. This is not only inconvenient and irritating, but it also drives up the cost of healthcare. Due to peripheral vascular damage and inadequate glucose management, diabetic patients are more likely to experience abnormal wound healing. The development of new drugs is urgently needed to address the drawbacks of existing ones [23].

The dermis, epidermis, and subcutaneous fat must work in concert to restore the skin. The external environment is too harsh for the epidermis to withstand [24]. As a result, the human body is exposed to a hostile external environment, including the invasion of germs and other diseases, after the epidermis is destroyed. Antimicrobial medications should be added to dressings during this process. Extracellular stromal immune cells, etc., are abundant in the dermis and may offer immunity and nourishment [25]. The dermis still receives growth hormones from subcutaneous fat. Hypoglycemic medications can be utilized for glycemic management to lower glucose levels at the wound site since the dermis has a large number of capillaries. The stages that are typically seen in a wound that is healing normally are hemostasis, inflammation, proliferation, and remodeling [26].

Hyperglycemia and redox imbalances (oxidative stress and decreased tissue antioxidant capacity) may cause neuropathy or ischemic lesions, in addition to hindering the healing of diabetic wounds [27]. Reductants, which are naturally occurring substances that effectively remove oxidizing agents like ROS, shield the body from harm. The rate of wound healing is also influenced by its pH, and the normal pH range of skin is approximately 5.5. Due to increased blood flow, wounds connected to diabetes have an elevated pH (pH of 7–9) [28], which not only irritates the wound but also encourages the growth of germs. Thus, altering the pH value is also required to hasten the healing of wounds. Alternatively, the hydrogel's pH-specific response can be enhanced by the wound's high pH, promoting the spread of active gradients.

## 4 Bioactive compounds in wound healing

Bandages with antioxidant, anti-inflammatory, and antibacterial qualities are believed to be "ideal" for treating chronic wound problems and encouraging acute wounds to heal normally. Numerous studies have already demonstrated the positive effects of the bioactive chemicals produced by cyanobacteria on skin [1,29]. Because of the many therapeutic benefits of *Spirulina platensis*, also known as *Arthrospira*, societies in Africa, Mexico, and the Far East have used it as a nutritional supplement since ancient times. Compounds from *S. platensis* formed from various extracts have the ability to speed up wound healing, while the underlying mechanisms are still need to be understood. Research has also revealed that the *S. platensis* extracts had no cytotoxic effects on fibroblasts or human peripheral blood cells [29].

An *in vitro* scratch assay revealed an increased closure rate of the wound area within 24 h of treatment, proving that *S. platensis* aqueous extract stimulate cell proliferation and migration at low doses (50 μg/ml) to accelerate wound healing [30]. Additionally, topical application on burned and injured rats resulted in the downregulation of fibrotic genes (*TGF-β1* and *α-SMA*) and the upregulation of angiogenic genes (*bFGF* and *VEGF*). At doses of 0.5 % and 1.125 % of crude extracts, *in vitro* wound-healing experiments demonstrate an increase in cell migration and proliferation from 23 % to 56.6 % and 74.9 %, respectively. *S. platensis* extracts have also been used in the context of cosmetic development to formulate a skin cream for the treatment of skin injuries. Immunohistochemistry studies revealed that adding skin cream extract increased the amount of collagen I deposition by 0.5 % and 1.125 % [31].

Among the most prevalent illnesses brought on by these resistant bacteria are infections of the skin and soft tissues. Vancomycin was discovered to be masked by *Chlamydomonas reinhardtii*, and its release required the insertion of a photocleavable linker. When this living pharmaceutical carrier was tested in *Bacillus subtilis*, UVA1-mediated release was the sole technique to halt the bacteria's growth. These findings are among the first instances of medication delivery for UVA1-induced antibiotic release through a living creature [32].

Obaíd et al. [33] suggested that photosynthetic cells may be implanted to deliver oxygen to organs in the case of a lack of arterial supply. While several *in vitro* and *in vivo* models have demonstrated the potential of this approach, its safety in actual patients remains unclear. This early phase 1 clinical study is evaluating the safety and viability of implanting photosynthetic scaffolds for dermal regeneration in eight individuals with full-thickness skin lesions. Overall, this work shows that the photosynthetic microalgae *Chlamydomonas reinhardtii* present in the implanted scaffolds did not induce any adverse local or systemic immunological reactions, and over a ninety-day period, they supported complete tissue regeneration in persons (Fig. 2).

**Fig. 2:** Microalgal based implanted scaffold. Preparation of wound bed for scaffold implantation (A). Photosynthetic scaffolds sutured on the wound (B,C), and covered with a polydimethylsiloxane membrane (D), followed by securing with negative pressure wound therapy and placement of light device on top (E,F). Adapted with permission from Ref. [33].

In a past study, the impact of sacran hydrogel film (Sac-HF) containing EGF, named as Sac/EGF-HF on *in vitro* cell migration utilizing a fibroblast cell line was demonstrated. The uniform Sac/EGF-HF film produced by the casting process was confirmed by morphological investigation. Additionally, after adding EGF, Sac/EGF-HF demonstrated notably increased thickness, tensile strength, and degradability. The higher mechanical strength of Sac/EGF-HF (3.8 MPa) in comparison to that of Sac-HF (1.7 MPa) proved the durability of HF. Sac/EGF-HF had a reduced ability for swelling in comparison to Sac-HF; supporting the tensile strength outcome. Remarkably, the differential scanning calorimetry and X-ray diffraction data for Sac/EGF-HF revealed an amorphous structure. According to the *in vitro* research, Sac/EGF-HF enhanced the migration of fibroblasts [34].

Recent research has focused on phytoconstituent-based therapies targeting the nuclear factor-kappa B (NF-κB) pathway, a key transcriptional factor in the healing process, supports diabetic wound healing. The study further examined papers from reliable databases such as Web of Science, EMBASE, Google Scholar, PubMed, Scopus, and Science Direct. Based on these investigations, the compounds found in plants included monoterpene glycosides, alkaloids, polyphenols, flavonoids, triterpenoids, and phenolics. The study was further concluded that the following agents show promise for the treatment of diabetic wound healing: Plumbagin, Berberine, Betulinic acid, Syringic acid, Loureirin-A, Gallo catechin, Loureirin-B, Paeoniflorin, Puerarin and Lupeol; Neferine, Boswellic acid, Plumbagin, Luteolin, Genistein, Rutin, Kirenol, Vicenin-2; Icariin, Gamma-tocopherol; Resveratrol. Numerous studies on various phytoconstituents have shown their influence on signaling pathways, such as NF-κB. These findings provide hope for the development of medicinal phytoconstituents to aid in the treatment of diabetic wounds that persist over an extended period of time [35]. Summary of the potential therapeutic wound healing chemicals derived from microalgae is shown in Fig. 3.

**Fig. 3:** Summary of the few potential therapeutic wound healing chemicals derived from microalgae. The illustration is based on the information published by Kanwal and De-Eknamkul [72], Kanwal and Incharoensakdi [73] and Kumar et al. [74] *GABA: γ-aminobutyric acid; ALA: δ-aminolevulinic acid; PUFAs: Polyunsaturated fatty acids.*

## 5 Microalgal wound healing

### 5.1 Hydrogel based wound healing

Hydrogels have been studied as novel adhesive materials with numerous applications. Hydrogels have the ability to stick to a wide range of surfaces, such as metals, polymers, biological tissues, and other hydrogels. Effective hydrogel adhesion can be challenging to achieve, though, it depends on specific binding and moisture levels. Furthermore, the adhesion of alginate gel and nanocomposite hydrogel has also been discussed [36]. To maximize the adhesion between the hydrogels, several factors influencing the peeling energy between the interfacial adherent hydrogels must be taken into account. For peeling behavior, three groups were found. Scanning electron microscopy (SEM) images and microscopy were used to confirm the establishment of a stable adherent contact. Moreover, elemental analysis using SEM-EDS was employed to investigate the hydrogel adhesion process. The effectiveness of interfacial adherent hydrogels in an aquatic environment was tested by conducting stability tests and experiments involving the immobilization of microalgae created a stable bond between the alginate gel containing microalgae and the nanocomposite hydrogel [36].

In a recent study by Chen et al. (2024)Chen et al. [37], improvement in the wound healing process in diabetic mice was noted in response to SIKVAV-modified chitosan hydrogels (Fig. 4). Chitosan hydrogels are considered suitable in tissue engineering due to their biocompatibility as well as non-toxicity and have also shown the great capacity of enhanced healing in irregular wounds [38]. Rozan et al. [39] enhanced wound healing by combining diatom biosilica (DBs) with doxycycline (DOXY) and coated them with hydroxybutyl chitosan (HBC) hydrogel. The HBC/DBs/DOXY composite hydrogel exhibited significant inhibitory effects on *S. aureus* (100 %) and *Escherichia coli* (98 %). Additionally, the HBC/DBs/DOXY hydrogel demonstrated minimal cytotoxicity on L929 cells *in vitro*, suggesting high biocompatibility. *In vivo* experiments indicated that the HBC/DBs/DOXY composite hydrogel may hasten wound healing and encourage re-epithelialization. Following a 12-day hydrogel treatment, 99.4 ± 0.4 % of wounds healed, indicating neovascularization and collagen deposition.

**Fig. 4:** Enhanced contraction of skin wounds in diabetic mice under application of SIKVAV-modified chitosan hydrogel. Typical wounds among the various tested groups (A) and statistical evaluation (B). Adapted with permission from Chen, Cao, Zhang, Jiang, Yu and Chen [37].

Kopač et al. [40] used a consistent 2 % alginate (w/v) and escalating concentrations of gelatin (w/v)) (up to 1 %) to encapsulate *Chlamydomonas reinhardtii*. The hydrogels were then crosslinked with a 0.43 % CaCl_2_ solution. This was done with the potential application of hydrogel patches in mind, as they can help oxygenate wounds to facilitate healing. The crosslink density of the hydrogel affected cell growth and oxygen production, considering their rheological properties. It was found that nutrient diffusion plays a key role in regulating cell proliferation and oxygen production within the encapsulated cells. It was demonstrated that changing the gelatin concentration could greatly regulate diffusion. The concentration of gelatin molecules increased once it was established that the gelation point was 0.66 % (w/v). At that point, oxygen production, cell development, and nutrient delivery were significantly impacted by the viscosity effect. On the other hand, crosslink density results in the creation of stable hydrogel networks at gel concentrations greater than the gelation threshold (up to 1 %), which influences nutrient transit, cell growth, and oxygen generation. In order to create alginate-gelatin systems with the best properties for a variety of applications, studies were done to find out how cell concentration affected the mechanical properties of hydrogels.

Using microfluidic electrospray technology, live hydrogel microspheres made of alginate filled with microalgae were successfully created to enhance wound healing. The combination of live alginate microspheres loaded with microalgae provides significant support for wound healing by ensuring excellent biocompatibility and effective oxygen release. Concurrently, the overall efficacy of wound treatment has enhanced due to the successful insertion of vascular endothelial growth factor (VEGF) into the microspheres. Coating the rat's wound with microalgae-VEGF-loaded alginate microspheres demonstrated significantly increased collagen deposition and vascular development during the wound closure process. Results showed that live alginate hydrogel microspheres containing microalgae are remarkably effective at accelerating the healing of wounds, opening up new avenues for future therapeutic treatment strategies [41].

Hydrogels are antimicrobial polymers that function as a physical barrier to retain moisture in the wound and prevent germs from entering. This makes them valuable for wound dressing treatments. They also exhibit superior mechanical and biocompatibility properties. Chitosan was combined with sulfated polysaccharides (PS) derived from three different types of red microalgae (freshwater, sea, and brackish) to create PS_sea/brackish/fresh_-Chi hydrogels. Further research revealed that PS/Chi hydrogels were the most rigid and stable under physiological conditions. The demonstrated properties of Zn-PS-Chi hydrogels have the potential to be used as wound dressings [42].

De Melo et al. [43] studied the evaluation of the hydrogel-based *C. vulgaris* extract's potential as an *in vivo* wound healing test was studied. Mice with excisional wounds were treated with a hydrogel formulation containing different amounts of extracts from *C. vulgaris* cultured in either mixotrophic or autotrophic conditions for 12 days. Tissue healing was assessed using macroscopic and histomorphometric methods. The antioxidant activity, hemagglutinating activity, protein content, phytochemical profile, and antibacterial activity of the extracts were determined using the DPPH (2,2-diphenyl-1-picrylhydrazyl) assay. Mice treated with hydrogel containing 25 % mixotrophic culture showed significant skin appendages, reduced fibroblast and inflammatory cell numbers, and increased collagen deposition in the wound-healing assay. Mixotrophic culture exhibited hemagglutinating activity ranging from ≥224 in human type B blood to ≥248 in rabbit erythrocytes, with a total protein content of 1.174 mg/ml. The phytochemical profile of the extract revealed the presence of sugars, triterpenes, steroids, and saponins. Additionally, mixotrophic culture demonstrated the highest levels of antibacterial activity (54.64 %) and antioxidant activity (54.64 %) against *Escherichia coli, Enterococcus faecalis*, and *Klebsiella pneumoniae*. The pro-healing and anti-inflammatory qualities of *C. vulgaris* cell extracts from mixotrophic culture were highlighted in this early investigation of a hydrogel formulation incorporating microalgae extracts for wound healing, which sped up the healing process.

Dried algal biomass, consisting solely of bioactive components, can be used with hydrogel scaffolds to enhance their antibacterial and wound-healing capabilities. This was achieved by creating algal biomass-loaded hydrogel scaffolds (AHS) from *Chlorella sorokiniana*. *C. sorokiniana* has been utilized in various settings over the years, sparking the interest of the pharmaceutical and cosmetic industries. Combining various phytochemicals and bioactive compounds has additional health benefits. Research to date has shown that AHS has potent anti-inflammatory and antibacterial properties, as well as accelerates wound healing. For 14 days, AHS (with various algal biomass concentrations) was topically applied to mice's excisional lesions. Wound healing was assessed using histology testing, microscopic inspection, and pro- and anti-inflammatory cytokine evaluations. Various methods, such as tests for swelling, rheology, temperature, and mechanical properties; Fourier transform infrared (FTIR); Raman; transmission electron microscopy; atomic force microscopy; X-ray diffraction; and SEM, were used to analyze and evaluate these scaffolds. AHS demonstrated significant biocompatibility and strong antibacterial efficacy against *Staphylococcus aureus* (98 %) and *Escherichia coli* (99 %). In addition to their antibacterial properties, the as-synthesized AHS may expand the range of effective wound healing techniques [44].

### 5.2 Nano based wound healing

Antimicrobial peptides are a novel class of drugs that have the potential to treat a variety of illnesses. Microalgal peptides from naturally occurring microalgae were electrospun with polycaprolactone (PCL) and κ-Carrageenan (κ-C) to produce nanofibers. SEM, fourier infrared spectroscopy, contact angle measurement and thermogravimetric analysis were used to investigate the peptides added to the nanofibers. The results showed that the wettability of nanofibers decreased upon the addition of peptides with molecular weights smaller than 10 kDa. The SEM investigation revealed thin, smooth, connected structures resembling beads. Using disc diffusion and minimum inhibitory concentration experiments against *Escherichia coli* (MTTC 443) and *Staphylococcus aureus* (MTTC 96), the antibacterial activity of the electrospun nanofibers was assessed. HEK 293 cell lines were used to confirm the produced nanofibers' *in vitro* biocompatibility, which exhibited a higher degree of cell viability of 98.32 % at 120 h. Remarkably, *in vitro* scratch tests demonstrated that the fibers exhibit remarkable wound-healing properties. The findings indicated that algal peptides and PCL/κ-C combined show antibacterial and biocompatible properties for use as biomaterials in wound healing procedures [45].

El-Baz et al. [46] reported that the green microalga *Dunaliella salina* is one of the primary sources of bioactive zeaxanthin and β-carotene. Therefore, studies on its antioxidant action in wound healing were carried out. The aim of those studies was to produce two novel products that were chitosan nanoparticles (CNPs)-loaded *D. salina* methanol extract (ME), named as ME-CNPs and hexane:ethyl acetate extract (HEAE) named as HEAE -CNPs for *in vivo* wound healing. The *in-vitro* release and *in-vivo* wound healing ability of the produced ME-CNPs and HEAE-CNPs were assessed in Wistar rats. The HPLC studies showed that HEAE of *D. salina* comprised 16.196 mg/g of zeaxanthin and 19.167 mg/g of β-carotene, while the ME has far less zeaxanthin (0.313 mg/g). Both HEAE-CNPs and ME-CNPs showed signs of wound healing and regeneration by downregulating tumor necrosis factor alpha and upregulating collagen skin contents as well as VEGF.

### 5.3 Bioactive compounds in wound healing

Miguel et al. [47] explored the potential advantages in wound-healing applications that have been connected to the diverse biological activities of PUFAs, polysaccharides, microalgal carotenoids, and crude extracts. ROS are quenched, inflammatory cytokine and transduction cascade generation are suppressed, and microbial growth at the wound site is prevented, among other actions. In order to cure skin damage, an evaluation of microalgae-based wound dressings and their bioactive ingredients is done. Finally, novel methods for producing living microalgal-based photosynthetic scaffolding for skin regeneration are also discussed. Bioactive compounds extracted from microalgae for utilization in diabetic wound healing are shown in Table 1.

**Table 1:** Bioactive compounds extracted from microalgae for utilization in diabetic wound healing.

**Bioactive compounds**	**Nature of chemical compound**	**Effects on Diabetes Mellitus Wound Healing**	**References**
Chlorella growth factor (CGF)	A complex mixture of various substances extracted from *Chlorella* (nucleic acid, amino acid, peptide, vitamins and polysaccharide)	- cellular regeneration - ↑support the regeneration of skin cells - ↑cell regeneration - ↑inflammatory cells that support the speed of wound healing	[75]
Astaxanthin	A carotenoid derived from microalgae	- inhibits the expression of inflammatory cytokines (COX-2, TNF-α, IL-6, and IL-1β)	[63,[76], [77], [78], [79], [80], [81], [82]]
β-Carotene	A carotenoid precursor to vitamin A	- ↑increases the tissue integrity - ↑defenses cell activity	[49,75]
Phycobilin	A pigment found in cyanobacteria and red algae	- ↑angiogenesis - ↑collagen synthesis	[75,83]
Chlorophyll *a*	A photosynthetic pigment integral to the primary light-capturing reactions in plants, algae, and cyanobacteria	- ↓TNF-α - ↓IL-1β - ↓IL-6 - ↑IL-10 - ↑TGF-β	[49,75,[83], [84], [85]]
Phycocyanin	A protein-bound pigment involved photosynthetic light capture and radical scavenging	- ↑fibroblast proliferation - ↑induced cellular migration to recover wound area	[49,83]
Allophycocyanin	A phycobiliprotein facilitating energy transfer in photosynthetic complexes of cyanobacteria and red algae	- ↑oxygen delivery to the wound site - ↑promoting cell growth	[49]
Phenolic compound	A diverse class of secondary metabolites	- antioxidant activities that help in reducing oxidative stress during wound healing	[49]
Flavonoids, alkaloids, and triterpenoids	Bioactive phytochemical compounds	- antimicrobial and wound contraction property - ↑increased rate of epithelization	[83]
Polysaccharides and exopolysaccharide	High-molecular-weight carbohydrates involved in structural integrity, hydration, and biofilm formation	- ↑collagen synthesis - ↑angiogenesis	[49,67,[86], [87], [88], [89], [90]]
Xylan and Carrageenan	Plant- and algae-derived polysaccharides	- ↓reduced inflammation - ↑scratch-wound healing - ↑stimulated cell proliferation - ↑TGF-β1 expression - ↑anti-coagulation activity	[89,91]
Alginate	A polysaccharide extracted from brown algae	- increase in the number of fibrocytes, fibroblasts, and macrophages - increase the percentage of collagen densities - decrease the number of neutrophils - activating Nrf2 - promotes angiogenesis via upregulation VEGF expression - ↑blood clotting	[[91], [92], [93], [94]]
β-Glucans and Paramylon	Glucose polymers	- ↑enhanced the activity of immune cells, such as macrophages and neutrophils - ↑production of growth factors - antioxidant activity	[[95], [96], [97], [98]]
Fucoidans	Sulfated polysaccharides from brown algae	- ↓ Matrix metalloproteinases	[91,99]
Essential fatty acids	Long-chain polyunsaturated fatty acids required for membrane fluidity and the synthesis of signaling molecules	- ↑angiogenesis - ↑collagen fiber formation and epidermis creation - controlling neutrophil migration and cytokine production	[49,52,100]
Triterpenes	Secondary metabolites contributing to membrane stability and signaling cascades	- *anti*-inflammatory properties that can speed up the healing process. - ↑collagen deposition, a decrease of fibroblast and inflammatory cells, strong evidence of skin appendages, and evidence of basal laminae	[43,49,96]
Lectins	Glucose polymers	- ↑promoting re-epithelialization and collagen deposition - ↑inducing immune system cells in the inflammatory phase resulting in the modulation of growth factors and cytokines - ↑stimulating collagen synthesis by fibroblasts and their differentiation	[49,101,102]

*Chlamydomonas reinhardtii*, a photosynthetic microalga, was encapsulated in alginate hydrogels and demonstrated good integration and rapid oxygen release when illuminated. Furthermore, the photosynthetic hydrogel demonstrated exceptional biocompatibility both *in vitro* and *in vivo*, in addition to its ability to maintain the oxygen necessary for the metabolic activities of skin explants and zebrafish larvae. ISO 10993–10:2010 parameters were used to evaluate photosynthetic dressings on twenty healthy human participants. The outcomes showed that the photosynthetic microalgae persisted in their survival and that the dressings did not irritate the skin. Additionally, antibiotics or genetically altered microalgae that release human VEGF were pre-loaded into hydrogels. The outcomes showed that both of the bioactive substances were continuously released. Overall, it is a feasible approach to locally distribute oxygen and bioactive compounds using photosynthetic hydrogels to promote wound healing [48].

de Andrade et al. [49] discussed that both *Chlorella* and *Spirulina* appear to be promising cyanobacteria due to their triterpenes, sugars, phenols, as well as proteins like phycocyanin and lectins. Zen Nutrients, WoundVite® (A *Chlorella* based nutritional supplement) claims to help with wound healing, scar reduction, and post-surgical recovery [50]. An alginate based wound dressing “3M™ Tegaderm™” is also commercially available [51]. However, little is known about the specific function and nature of the targeted bioactive compounds on the skin. Many microalgae and cyanobacteria genera have been reported to contain high amounts of pigments such hydroxypheophytin, chlorophyll *a*, β-carotene, and allophycocyanin; however, their effects on the different stages of wound healing are unknown. Developing innovative topical drugs from photosynthetic microbes is another practical way to aid in the healing process.

### 5.4 Fatty acids in wound healing

The antioxidant characteristics of the extracts and the effectiveness of fatty acid extraction from *Parachlorella kessleri* microalgae in the treatment of burns and excisional wounds were studied previously [52]. The importance of fatty acids in membrane phospholipids and their role in the inflammatory response justifies the investigation. Based on the 50.38 % increase in the percentage of PUFAs in the glycine culture of *P. kessleri*, it showed higher antioxidant and DPPH radical scavenging activity than that of the control. After being put under anesthesia, thirty male mice were split into six groups and used to either burn or excise two comparable full-thickness skin lesions paravertebral. Mice with excision wounds received twice-daily treatments with *P. kessleri* oils (extracted from glycine and control cultures) or the vehicle, placebo cream. *P. kessleri* oil and placebo cream were used in the treatment of burn patients. Both the control and glycine culture *P. kessleri* oils significantly reduced burns and excisional wounds. Angiogenesis, collagen fiber development, and epidermis creation were among the healing signs that improved, according to histopathological investigation.

### 5.5 Polysaccharides in wound healing

An *in vitro* study by Tseng et al. [53] evaluated the anti-allergic and wound-healing properties, safety, and biochemical makeup of *Nostoc* commune polysaccharide-rich extract. Elements (Ni, Ba, Mn, Sr, and K) and bioactive chemicals (total phenolic, total flavonoids, and sulfates) were found highly concentrated in the extract. Glucose makes up the bulk of the extract's 221.69 ± 25.56 mg/g polysaccharide. Tests for heavy metals and cytotoxicity verified the extract's safety and availability. In cell culture studies, the polysaccharide effectively inhibited β-hexosaminidase and IL-6, while simultaneously inducing the production of collagen I. These findings suggested that the extract could be a useful ingredient in cosmetics that heal wounds and reduce allergies.

In another study, Alvarez et al. [54] investigated the exopolysaccharides (EPS) generated by the strains of *Nostoc* sp. PCC7936 and PCC7413 and assessed as possible biomaterials for novel wound dressings. The amount of EPS produced was marginally increased up to 1463.1 ± 16.0 mg/l (PCC7413) and 1372.1 ± 29.0 mg/l (PCC7936), by adding acetate ions to the growth media. The anionic character and the presence of sulfate groups in both EPS—critical characteristics for biomedical applications—were confirmed by FTIR and dynamic light scattering data. It was further noted that in the presence of 0.4 % (w/v) FeCl_3_, both EPS at 1 % (w/v) were able to form gels. Results from the 3-(4,5-dimethylthiazol-2-yl)-2,5-diphenyl tetrazolium bromide colorimetric assay and *in vitro* scratch assays suggested that PCC7936 derived hydrogel was more biocompatible and could encourage fibroblast migration and proliferation.

### 5.6 Phytochemicals in wound healing

Rich in carotenoids, *D*. *salina* was studied for possible antagonistic effects on the structural and functional aspects of rats' thioacetamide (TAA)-induced hepatic fibrosis [55]. For six weeks, adult male albino Wistar rats were given TAA injection in addition to three dosage levels of *D. salina* extract or powder. The following enzyme levels were measured in serum: alkaline phosphatase, albumin, bilirubin, bilirubin, aspartate transaminase, and alanine transaminase. The liver's contents were also measured for reduced glutathione, collagen I, malondialdehyde, and smooth muscle actin alpha (α-SMA). Hepatic collagen I, α-SMA, aspartate transaminase, alanine transaminase, alkaline phosphatase and malondialdehyde levels were significantly reduced after treatment with *D. salina* powder or extract. Glutathione hepatic levels and serum albumin levels both showed notable rises. *D. salina* also decreased TAA-induced fibrosis, centrilobular necrosis, and inflammatory cell infiltration, according to a liver histology investigation. The outcomes showed that *D. salina* protects the livers of rats against TAA-induced fibrosis. A high quantity of total carotenoid (15.2 % of the algal extract) and other unsaturated fatty acids, like alpha-linolenic acid, have hepatoprotective effects, according to the phytochemical analysis.

Due to the potential risks associated with artificial coloring, natural coloring has become more and more popular in food and medicine. Because of its therapeutic and medical properties, phycocyanin is considered the most favored phycobilin pigment of the cyanobacterium *S. platensis*. Zamani et al. [56] used five freezing/thawing cycles, ultrasonic disruption, ammonium sulfate precipitation, and dialysis to extract and purify phycocyanin from *S. platensis.* Mice infected with *Candida albicans* were used to test the efficacy of phycocyanin-produced cream (containing 1.5 % and 3 % of phycocyanin in comparison to control) to confirm that phycocyanin has antifungal capabilities. The mice groups treated with the phycocyanin-containing formulation improved noticeably more quickly than the control group, according to the data.

An *in vitro* wound scratch test and three antioxidant assays were used to evaluate the *Nostoc* NIES-2111_MUM004 water extracts' capacity to accelerate wound healing [57]. In the tests of ferric reducing antioxidant power, β-carotene bleaching, and 2,2′-azino-bis (3-ethylbenzothiazoline-6-sulfonate radical scavenging, the water extracts showed good antioxidant characteristics and a high protein content. Furthermore, the findings of the cytotoxicity assay showed that extracts could be used safely up to 250 μg/ml. Water extracts at 125 μg/ml demonstrated significant migration and proliferation activity, with 42.67 % of wounds closed. It was determined that phycobiliproteins were not the only one in charge of wound healing activities when statistical correlation showed no significant association (*p>0.05*) between the protein fraction and the wound healing characteristics. Prioritizing these results is crucial for identifying reliable providers of bioactive compounds from innovative and sustainable sources, ultimately expanding the application of microalgae in the fields of nutrition, medicine, and cosmeceuticals.

Gunes et al. [58] found that after three days, the 0.1 % *S. platensis* extract showed higher proliferative activity than the control group, with 198 % of the cells still alive. When skin cream containing 1.125 % *S. platensis* crude extract was applied, the HS2 keratinocyte cell line showed better wound healing features; this concentration also produced the highest HS2 cell viability percentage. Creams containing *S. platensis* extract did not cause genotoxicity in human peripheral blood cells, according to the micronucleus experiment. Immunohistochemical tests revealed that collagen 1 immunoreactivity was significantly positive in cells treated with skin cream containing 1.125 % extract emphasizing that increased extract concentration can enhance collagen 1 immunoreactivity. Studies on genotoxicity, wound healing activity, and cell viability suggested that skin cream containing *S. platensis* may find use in the biological and cosmetic sectors.

## 6 Microalgal diabetic wound healing

### 6.1 Hydrogel in diabetic wound healing

Using a bioactive hydrogel technology, Hu et al. [59] developed a multifunctional quorum sensing (QS) inhibitor that decreases hypoxia, breaks down biofilms, and inhibits bacterial growth. In diabetic mice, this inhibitor also accelerates the healing of infected wounds. They loaded berberine (BBR), an antibacterial and QS inhibitor, into the naturally occurring microalgae *S. platensis* along with carboxymethyl chitosan/sodium alginate to form a bioactive hydrogel called BBR@SP gel. When exposed to laser light, the BBR@SP gel may continuously release BBR and generate ROS. In combination with chemo-photodynamic therapy for methicillin-resistant *Staphylococcus aureus*, this would disrupt QS. Additionally, the BBR@SP gel inhibits the production of virulence factors and stops and destroys the formation of biofilms (>82 % destruction rate). It was found that the BBR@SP gel could speed up the healing of diabetic wounds infected with methicillin-resistant *Staphylococcus aureus* by inducing angiogenesis, promoting skin regeneration, and lowering the inflammatory response. The wound closure rate was enhanced up to ∼98.4 % under the application of BBR@SP in combination with laser. Through a synergistic chemo-photodynamic mechanism, this research provides a novel antibacterial method that lowers biofilm hypoxia, suppresses QS, and kills drug-resistant bacteria. This strategy might provide fresh perspectives in the battle against illnesses linked to biofilms and antibiotic drug resistance.

An oxygen-producing patch that can generate dissolved oxygen was described in a study report [60]. The hydrogel used in its formulation is made from living microalgae. The patch worked more than 100 times better than topical gaseous oxygen, which penetrates the skin, as it distributes dissolved oxygen into the skin. Further studies suggest that the patch may improve the survival of skin grafts in diabetic mice as well as the healing of chronic wounds. Additionally, it might promote *in vitro* tube formation, cell motility, and proliferation. Because the microalgae-gel patch continually provides dissolved oxygen, it can effectively aid in the healing of chronic wounds.

A novel three-functional microalgae gel has been created by Jin et al. [61] and is intended for use in the treatment and management of chronic diabetic ulcers. The covalent organic framework (COF) modifies the gel. The gel is composed of a COF that reacts to ROS and a microalgae matrix that releases basic fibroblast growth factor (bFGF). While studies have suggested that two of these elements might aid in wound healing, combining all three roles offers a novel way to enhance the management of diabetic chronic wounds. Consequently, a novel notion known as "ligand interlocking" was introduced, offering three beneficial synergistic outcomes. In particular, the COF functions similarly to the "double Excalibur," which binds bFGF to stimulate angiogenesis and proliferation in chronic wounds, thereby inhibiting the inflammatory response. It also binds live microalgae to remove ROS and release dissolved oxygen to relieve wound hypoxia. Moreover, RNA sequencing analyses and *in vivo* experiments demonstrated that the COF-modified microalgae gel improved vascular and tissue regeneration at the wound site by blocking the inflammatory cascade cycle. The COF-modified microalgae gel is a potential technique for the active *in vivo* delivery of medication to the wound body in an intensive care unit scenario.

Wu et al. [62] reported that the diabetes patients need oxygen and electrical stimulation to encourage cell migration and differentiation in order to treat chronic wounds and restore damaged tissues. Although the medical community is widely aware of *Chlorella'*s great oxygen-generating capacity, not much research has been done on the possible applications of extracellular electron production for skin regeneration, that led to the development of sodium alginate and polyacrylamide (CHPS) hydrogels, which are semi-permeable networks of *Chlorella*. Acrylamide crosslinks due to free radicals, creating this network, which is then covered in chains of alginate. CHPS hydrogels effectively protect wounded tissue, provide *Chlorella* with mechanical support against external stimuli, and establish the perfect artificial microenvironment for *Chlorella* growth when applied to wounds. CHPS hydrogels exhibited impressive adhesion properties and fracture elongation, continuously generating oxygen and photosynthetic bioelectrical currents. Furthermore, angiogenesis, migration, and cell proliferation are all significantly improved by the extended release of bioelectricity and dissolved oxygen (with dissolved oxygen concentration ∼4 mg/l/h) by CHPS hydrogels, which enhances wound healing in diabetic mice. These results strongly support further investigation into CHPS hydrogels as a readily available, reasonably priced, and low-risk strategy to enhance the clinical care of diabetic patients with chronic wounds.

Kang et al. [63] studied the possibility of bacterial invasion, a complex inflammatory milieu, increased ROS, and acute hypoxia, diabetic wounds carry a lifelong risk of developing into diabetic foot ulcers. Here, a structured course of therapy is established using live *Haematococcus* (HEA). HEA has potential for use in programmed therapy since it can be programmed to carry out a variety of tasks by varying the intensity of the light. These tasks include the transfer of oxygen, the scavenging of ROS, immunological control, and antibacterial activity. Green HEA (GHEA), which has effective photothermal conversion at high light intensity (658 nm, 0.5 W/cm^2^), mediates wound surface disinfection. The photosynthetic system of GHEA is able to constantly create oxygen by lowering the light intensity (658 nm, 0.1 W/cm^2^), which fixes the hypoxia problems and encourages vascular regeneration. When HEA cells are exposed to continuous light, astaxanthin builds up, and the cells gradually change from green to red HEA. The ability of the living HEA hydrogel to promote cell migration and proliferation, speed up neoangiogenesis, and accelerate diabetic wound healing in female mice appears promising.

Hydrogels of *Chlorella* sp. were created by Wu et al. [64] to treat diabetic lesions. *In vitro* experiments showed that living *Chlorella* could actively consume glucose, create dissolved oxygen through photosynthesis, and use its inherent antioxidants to lower ROS throughout the day. Chlorine dioxide was utilized to inactivate the bacteria *in situ* at night at a concentration suitable for human health to take advantage of its abundant components. Studies conducted *in vitro* have demonstrated that inactivated *Chlorella* can nourish, reduce inflammation, and prevent the respiration of oxygen-using *Chlorella. Chlorella's* components and advantages as a living creature were expertly blended. It has been demonstrated that the previously indicated mechanisms accelerate angiogenesis, migration, and cell division *in vitro*. For additional validation, streptozotocin-induced diabetic mice were used. The results obtained *in vivo* validated that *Chlorella*, when combined with other elements, might improve tissue regeneration by reducing detrimental microenvironments such as elevated hyperglycemia, low oxygen levels, high ROS, and persistent inflammation. These results suggested that *Chlorella* is a specially designed treatment approach for the healing of diabetic lesions.

A hydrogel that continuously produces hydrogen for 60 h was demonstrated by Chen et al. [65] It is made up of bacteria and live *Chlorella* enclosed in a shell that is resistant to cells. This microbe-hydrogel system can minimize inflammation and toxic •OH and ONOO-species with selectivity. More research indicates that the microbe-hydrogel patch may promote cell proliferation and speed up diabetic wound healing by about 50 % on day three. Because of its exceptional biocompatibility and capacity to scavenge ROS, the hydrogel incorporating symbiotic bacteria and algae has significant promise for therapeutic application.

### 6.2 Microbot technology in diabetic wound healing

Many platforms have been developed to modify the immune response and/or reduce hypoxia to treat diabetic chronic wounds. However, the passive diffusion of therapeutic chemicals through the blood clot may be the reason for the rather poor delivery efficacy of these platforms to the deep wound site. A biohybrid microrobot based on microalgae was developed for diabetic wound healing. The biohybrid microrobot generated oxygen to treat hypoxia while moving autonomously at a speed of 33.3 μm/s. To control immunological responses, the microrobot also successfully bound to inflammatory chemokines such as interleukin-8 and monocyte chemoattractant protein-1. The enhanced retention and penetration of the microrobot in the skin tissue of a real wounded mouse are demonstrated by detecting fibrin clots in a biomimetic wound using microfluidic devices. After nine days, diabetic mice with chronic wounds that were treated with microrobots without the need for wound dressings fully recovered. Significant increases in angiogenesis—which exceeded 20 times the number of CD31^+^ cells—and a sharp decline in inflammatory cytokines—which dropped to less than 31 % of the control level—served as evidence for this. These results lend credence to the feasibility of utilizing microrobots as an innovative platform for diabetic wound care [66].

### 6.3 Polysaccharides in diabetic wound healing

Chitosan sponges were created and assessed by Vazquez-Ayala et al. [67] for use as wound dressings. The sponges were administered fucoidan, metformin, and EPS from *Porphyridium purpureum* algae, which are the medications being studied for potential medicinal applications. The mechanical investigation indicated that sponge composites, especially those with compressive strengths more than 30 kPa, exhibited good mechanical performance and shape memory under compression stress. These findings were associated with the porosity of the materials, which affected the swelling capacity, which peaked at 70 %. The material's shape was examined using SEM, and folded films with surface porosity were found. The biocompatibility testing findings showed that the materials have excellent antibacterial activity and are neither cytotoxic nor hemolytic. Metformin-loaded chitosan sponges were found to regenerate skin tissue over the course of a 21-day treatment period in the evaluation of *in vivo* wound healing. Histological investigations supported this conclusion, which highlighted the rapidity of healing that happens when EPS are administered to promote tissue regeneration. These results suggested that chitosan sponge compounds could be used as diabetic foot wound dressings. The microalgal originated polysaccharides are well desired for developing wound dressing such as hydrogels and films, due to their biocompatibility. Also, providing a moist environment at wounded site by imposing low toxicity makes them effective for utilization in wound dressings [68]. Fig. 5 summarizes the potential pharmacological wound healing applications derived from various algal groups.

**Fig. 5:** Potential pharmacological applications of various algal groups in wound healing.

### 6.4 Phytochemicals in diabetic wound healing

In an effort to accelerate the healing of diabetic wounds, Hussein et al. [69] studied the use of an algal extract primarily composed of *Microcystis aeruginosa* in the formulation of medicated bandages. Astaxanthin, phytoene, and hydroxypheophytin-*a* were the components of the algal extract identified and extracted after a phytochemical examination. These substances exhibited potent antioxidant and anti-inflammatory effects at 500 mg/kg. At 200 and 400 mg/kg, they significantly and dose-dependently reduced the glucose levels in the plasma of diabetic rats. The serum levels of insulin, glucose transporter 2, and cluster of differentiation 4 were much higher compared to catalase and nitric oxide. The results indicated that diabetic rat wounds treated with medicinal bandages made from algae healed more slowly than rats without treatment and exhibited lower tumor necrosis factor-α serum levels than collagen I levels.

### 6.5 Bioprinting scaffolds in diabetic wound healing

The 3D bioprinting is a cutting-edge technology that makes possible layer-by-layer printing of biological materials, including cells, biomaterials, and growth factors, to create 3D structures resembling tissues or organs. It holds significant promise in areas like tissue engineering, regenerative medicine, and drug testing and has the potential to reshape medicine by enabling the creation of human tissues and organs, making drug testing more accurate, and advancing the personalized treatment options [70]. Wang et al. [71] created a novel live photosynthetic framework that enables *in situ* microfluidic assisted 3D bioprinting to promote healing in wounds with uneven shapes. The method was inspired by the symbiotic relationship that exists naturally between salamanders and algae. The sustainable synthesis of oxygen under light irradiation was made possible by the insertion of *Chlorella pyrenoidosa*, a unicellular microalga that photosynthesizes oxygen, inside the 3D printed scaffolds. This made it possible to support cell motility, proliferation, and differentiation even in environments with low oxygen levels. Therefore, by reducing local hypoxia, boosting angiogenesis, and encouraging the production of ECM, living microalgae-laden scaffolds may be directly printed into diabetic wounds to dramatically speed up the chronic wound closure process. The study's findings implied that living photosynthetic microalgae can be bioprinted *in situ* to create an efficient autotrophic biosystem for wound healing, providing a therapeutic option for a range of tissue engineering applications.

## 7 Challenges

Microalgae hold significant potential for enhancing wound healing, particularly in the context of diabetic wounds. However, several challenges must be addressed to fully realize their therapeutic potential. First, the complex nature of the wound healing process, involving various cell types and biochemical interactions, makes it difficult to integrate microalgae effectively. Additionally, there is a lack of comprehensive understanding regarding the composition and mechanisms of action of microalgae, which hinders their widespread use in clinical practice [62]. While some research has explored the therapeutic effects of microalgae, more extensive studies are needed to evaluate their efficacy and safety, especially through randomized controlled trials [35]. These trials are crucial for determining microalgae's ability to prevent diabetic wounds and reduce the risk of complications such as amputations [59]. Translating laboratory findings into practical, clinically approved treatments poses additional challenges, including scalability, safety, and regulatory approval. Ethical concerns about sourcing and processing microalgae further complicate their adoption. Finally, integrating microalgae-based treatments into mainstream clinical practice requires global collaboration, regulatory approval, and extensive research to develop feasible, personalized treatments [59]. Overcoming these challenges will be crucial in advancing microalgae as a viable option for diabetic wound healing and other therapeutic applications.

## 8 Conclusion and prospect

In summary, microalgae derived bioactive compounds and metabolites have potential pharmaceutical applications in diabetic wound healing processes. The existing scientific literature emphasizes the utilization of microalgal biometabolites as alternative therapeutic approach for not merely due to their efficacy but also owing to their substantial contribution to the sustainability approaches. While there are few studies that have explored the potential of using microalgae to enhance diabetic wound healing, many have examined the therapeutic effects of algae. It is therefore essential to investigate the use of microalgae to prevent diabetic wound healing from occurring in the first place and later on to reduce the risk of amputations. There is no longer any excuse for not conducting randomized controlled trials on the preventive use of microalgae in a therapeutic setting for individuals at high risk of developing diabetic sores. To oversee a significant clinical trial, monitoring the occurrence and recurrence of diabetic wound healing, as well as the treatment's effectiveness and any negative impacts on the risk-benefit ratio, is crucial. However, more research is needed in this area as the literature has not focused much on the role of bioactive molecules in diabetic wound healing. Extensive preclinical and clinical research, regulatory approval and global collaboration procedures are necessary to integrate microalgae-based treatments into mainstream clinical practice and provide a feasible path toward more personalized and effective diabetic wound healing treatments.

**Table:** List of abbreviations

**PUFAs**	Polyunsaturated fatty acids
**ROS**	Reactive oxygen species
**3D**	Three-dimensional
**ECM**	Extracellular matrix components
**α-SMA**	Smooth muscle actin alpha
**h**	Hours
**PCL**	Polycaprolactone
**κ-C**	κ-Carrageenan
**AHS**	Algal biomass-loaded hydrogel scaffolds
**FTIR**	Fourier transform infrared
**CNP**	Chitosan nanoparticles
**COF**	Covalent organic framework
**bFGF**	Basic fibroblast growth factor
**CHPS**	Sodium alginate and polyacrylamide
**HBC**	Hydroxybutyl chitosan
**DBs**	Diatom biosilica
**DOXY**	Doxycycline
**TAA**	Thioacetamide
**DPPH assay**	2,2-Diphenyl-1-picrylhydrazyl assay
**EPS**	Exopolysaccharides
**HEAE**	Hexane:ethyl acetate extract
**ME**	Methanol extract
**NF-κB**	Nuclear factor kappa-B
**PS**	Sulfated polysaccharides
**BBR**	Berberine
**Sac/EGF-HF**	Sacran/Epidermal Growth Factor-Hydrogel Film
**UVA**	Ultraviolet
**VEGF**	Vascular endothelial growth factor

## CRediT authorship contribution statement

**Jinjin Pei:** Writing – original draft, Visualization, Software, Resources, Methodology, Data curation. **Simab Kanwal:** Writing – review & editing, Writing – original draft, Visualization, Validation, Supervision, Software, Resources, Project administration, Methodology, Investigation, Data curation, Conceptualization. **Ramachandran Sivaramakrishnan:** Writing – original draft, Visualization, Validation, Supervision, Resources, Methodology, Investigation, Data curation, Conceptualization. **Kasinee Katelakha:** Writing – original draft, Methodology, Investigation.

## Declaration of competing interest

The authors declare that they have no known competing financial interests or personal relationships that could have appeared to influence the work reported in this paper.

## References

[1] Zhuang D., He N., Khoo K.S., Ng E.-P., Chew K.W., Ling T.C. (2022). Application progress of bioactive compounds in microalgae on pharmaceutical and cosmetics. Chemosphere.

[2] Del Mondo A., Sansone C., Brunet C. (2022). Insights into the biosynthesis pathway of phenolic compounds in microalgae. Comput. Struct. Biotechnol. J..

[3] Huang H., Lang Y., Zhou M. (2024). A comprehensive review on medical applications of microalgae. Algal Res..

[4] MacNeil S. (2007). Progress and opportunities for tissue-engineered skin. Nature.

[5] Ruseva K., Ivanova K., Todorova K., Vladov I., Nanev V., Tzanov T., Vassileva E. (2020). Antibiofilm poly(carboxybetaine methacrylate) hydrogels for chronic wounds dressings. Eur. Polym. J..

[6] Basha S.I., Ghosh S., Vinothkumar K., Ramesh B., kumari P.H.p., Mohan K.V.M., Sukumar E. (2020). Fumaric acid incorporated Ag/agar-agar hybrid hydrogel: a multifunctional avenue to tackle wound healing. Mater. Sci. Eng. C.

[7] Zeng Y., Zou R., Zhao Y. (2016). Covalent organic frameworks for CO2 capture. Adv. Mater..

[8] Zhang L., Liu M., Zhang Y., Pei R. (2020). Recent progress of highly adhesive hydrogels as wound dressings. Biomacromolecules.

[9] Khamaisi M., Balanson S. (2017). Dysregulation of wound healing mechanisms in diabetes and the importance of negative pressure wound therapy (NPWT). Diabetes Metabol. Res. Rev..

[10] Iravani S., Varma R.S. (2019). Plants and plant-based polymers as scaffolds for tissue engineering. Green Chem..

[11] Pillai M.M., Dandia H., Checker R., Rokade S., Sharma D., Tayalia P. (2022). Novel combination of bioactive agents in bilayered dermal patches provides superior wound healing. Nanomed. Nanotechnol. Biol. Med..

[12] Annabi N., Rana D., Shirzaei Sani E., Portillo-Lara R., Gifford J.L., Fares M.M., Weiss A.S. (2017). Engineering a sprayable and elastic hydrogel adhesive with antimicrobial properties for wound healing. Biomaterials.

[13] Sun B.K., Siprashvili Z., Khavari P.A. (2014). Advances in skin grafting and treatment of cutaneous wounds. Science.

[14] Fan Z., Zhu C., Yin J., Qin L., Zhao X. (2023). Pitaya-inspired microcarrier/hydrogel composite for chronic wound healing: one-pot preparation, tailorable structures, and versatile functionalization. Chem. Eng. J..

[15] Petkovic M., Sørensen A.E., Leal E.C., Carvalho E., Dalgaard L.T. (2020). Mechanistic actions of microRNAs in diabetic wound healing. Cells.

[16] Ge Y., Wang J., Cao W., Niu Q., Wu Y., Feng Y., Liu Y. (2022). Low temperature plasma jet affects acute skin wounds in diabetic mice through reactive components. Int. J. Low. Extrem. Wounds.

[17] Kolipaka T., Pandey G., Abraham N., Srinivasarao D.A., Raghuvanshi R.S., Rajinikanth P., Srivastava S. (2023). Stimuli-responsive polysaccharide-based smart hydrogels for diabetic wound healing: design aspects, preparation methods and regulatory perspectives. Carbohydr. Polym..

[18] Li D., Wu N. (2022). Mechanism and application of exosomes in the wound healing process in diabetes mellitus. Diabetes Res. Clin. Pract..

[19] Wu X., He W., Mu X., Liu Y., Deng J., Liu Y., Nie X. (2022). Macrophage polarization in diabetic wound healing. Burns & Trauma.

[20] Xu Z.-H., Ma M.-H., Li Y.-Q., Li L.-L., Liu G.-H. (2023). Progress and expectation of stem cell therapy for diabetic wound healing. World J. Clin. Cases.

[21] Azzari N.A., Segars K.L., Rapaka S., Kushimi L., Rich C.B., Trinkaus-Randall V. (2023). Aberrations in cell signaling quantified in diabetic murine globes after injury. Cells.

[22] Malissen B., Tamoutounour S., Henri S. (2014). The origins and functions of dendritic cells and macrophages in the skin. Nat. Rev. Immunol..

[23] Andonova M., Urumova V. (2013). Immune surveillance mechanisms of the skin against the stealth infection strategy of Pseudomonas aeruginosa—review. Comp. Immunol. Microbiol. Infect. Dis..

[24] Ginhoux F., Tacke F., Angeli V., Bogunovic M., Loubeau M., Dai X.-M., Merad M. (2006). Langerhans cells arise from monocytes in vivo. Nat. Immunol..

[25] Ronchese F., Hilligan K.L., Mayer J.U. (2020). Dendritic cells and the skin environment. Curr. Opin. Immunol..

[26] Rodrigues M., Kosaric N., Bonham C.A., Gurtner G.C. (2018). Wound healing: a cellular perspective. Physiol. Rev..

[27] Bolajoko E.B., Akinosun O.M., Khine A.A., Preedy V.R. (2020). Diabetes.

[28] Zhu Y., Zhang J., Song J., Yang J., Du Z., Zhao W., Zhang L. (2020). A multifunctional pro-healing zwitterionic hydrogel for simultaneous optical monitoring of pH and glucose in diabetic wound treatment. Adv. Funct. Mater..

[29] Lee J.-J., Kim K.B., Heo J., Cho D.-H., Kim H.-S., Han S.H., Bae S. (2017). Protective effect of Arthrospira platensis extracts against ultraviolet B-induced cellular senescence through inhibition of DNA damage and matrix metalloproteinase-1 expression in human dermal fibroblasts. J. Photochem. Photobiol. B Biol..

[30] Syarina P.N.A., Karthivashan G., Abas F., Arulselvan P., Fakurazi S. (2015). Wound healing potential of Spirulina platensis extracts on human dermal fibroblast cells. EXCLI journal.

[31] Gunes S., Tamburaci S., Dalay M.C., Deliloglu Gurhan I. (2017). In vitro evaluation of Spirulina platensis extract incorporated skin cream with its wound healing and antioxidant activities. Pharm. Biol..

[32] Shchelik I.S., Sieber S., Gademann K. (2020). Green algae as a drug delivery system for the controlled release of antibiotics. Chem. Eur J..

[33] Obaíd M.L., Camacho J.P., Brenet M., Corrales-Orovio R., Carvajal F., Martorell X., Egaña J.T. (2021). A first in human trial implanting microalgae shows safety of photosynthetic therapy for the effective treatment of full thickness skin wounds. Front. Med..

[34] Wathoni N., Rusdiana T., Hasanah A.N., Pratama A.R., Okajima M., Kaneko T., Arima H. (2020). Epidermal growth factor in sacran hydrogel film accelerates fibroblast migration. \"J. Adv. Pharm. Technol. Research\"\" (JAPTR)\".

[35] Yadav J.P., Verma A., Pathak P., Dwivedi A.R., Singh A.K., Kumar P., Patel D.K. (2024). Phytoconstituents as modulators of NF-κB signalling: investigating therapeutic potential for diabetic wound healing. Biomed. Pharmacother..

[36] Kim W.H., Han Y., Lee I.S., Won N.-I., Na Y.H. (2022). Development of hydrogel adhesion system for propagation of aquatic organisms. Polymer.

[37] Chen X., Cao X., Zhang J., Jiang C., Yu Y., Chen H. (2024). Enhancing skin wound healing in diabetic mice using SIKVAV-modified chitosan hydrogels. Journal.

[38] Mawazi S.M., Kumar M., Ahmad N., Ge Y., Mahmood S. (2024). Recent applications of chitosan and its derivatives in antibacterial, anticancer, wound healing, and tissue engineering fields. Journal.

[39] Rozan H.E., Wu G., Zhou Z., Li Q., Sharaf M., Chen X. (2022). The complex hydrogel based on diatom biosilica and hydroxybutyl chitosan for wound healing. Colloids Surf. B Biointerfaces.

[40] Kopač T., Boček Ž., van Midden K.P., Klemenčič M., Ručigaj A. (2023). Encapsulation of living photosynthetic organisms in alginate-gelatin hydrogels for controlled cell growth and oxygen production. Biochem. Eng. J..

[41] Jia J., Liu J., Shi W., Yao F., Wu C., Liu X., Liao Y. (2024). Microalgae-loaded biocompatible alginate microspheres for tissue repair. Int. J. Biol. Macromol..

[42] Netanel Liberman G., Ochbaum G., Bitton R., Arad S. (2021). Antimicrobial hydrogels composed of chitosan and sulfated polysaccharides of red microalgae. Polymer.

[43] de Melo R.G., de Andrade A.F., Bezerra R.P., Viana Marques D.d.A., da Silva V.A., Paz S.T., Porto A.L.F. (2019). Hydrogel-based Chlorella vulgaris extracts: a new topical formulation for wound healing treatment. J. Appl. Phycol..

[44] Agarwal A., Kumar A., Garg P., Chakraborty A., Verma R., Sarwat M., Mukherjee M. (2022). Algal biomass-loaded hydrogel scaffolds as a biomimetic platform with antibacterial and wound healing activities. ACS Appl. Polym. Mater..

[45] Raghunathan S., Kandasamy S., Balakrishna Pillai A., Senthilathiban D.P., Thajuddin N., Rasool Kamli M., Davoodbasha M. (2024). Synthesis of biocomposites from microalgal peptide incorporated polycaprolactone/κ- carrageenan nanofibers and their antibacterial and wound healing property. Int. J. Pharm..

[46] El-Baz F.K., Salama A., Ali S.I., El-Hashemy H.A. (2023). Dunaliella salina chitosan nanoparticles as a promising wound healing vehicles: in-vitro and in-vivo study. OpenNano.

[47] Miguel S.P., Ribeiro M.P., Otero A., Coutinho P. (2021). Application of microalgae and microalgal bioactive compounds in skin regeneration. Algal Res..

[48] Corrales-Orovio R., Carvajal F., Holmes C., Miranda M., González-Itier S., Cárdenas C., Egaña J.T. (2023). Development of a photosynthetic hydrogel as potential wound dressing for the local delivery of oxygen and bioactive molecules. Acta Biomater..

[49] de Andrade A.F., Porto A.L.F., Bezerra R.P. (2022). Photosynthetic microorganisms and their bioactive molecules as new product to healing wounds. Appl. Microbiol. Biotechnol..

[50] Zen nutrients https://zennutrients.com/products/woundvite?srsltid=AfmBOor6bK8OYX35_kfKYdlUvZj8RRuNHK3AVHbDbtks_gSTbsHATcua (accessed 8 January).

[51] 3M™ Tegaderm™ High Integrity Alginate Dressing https://www.3m.co.uk/3M/en_GB/p/d/b5005108002/. (accessed accessed 8 January).

[52] El-Sheekh M., Bedaiwy M., Mansour H., El-shenody R.A. (2024). Efficiency of the fatty acids extracted from the microalga Parachlorella kessleri in wound-healing. Burns.

[53] Tseng C.-C., Yeh H.-Y., Liao Z.-H., Hung S.-W., Chen B., Lee P.-T., Lee M.-C. (2021). An in vitro study shows the potential of Nostoc commune (Cyanobacteria) polysaccharides extract for wound-healing and anti-allergic use in the cosmetics industry. J. Funct.Foods.

[54] Alvarez X., Alves A., Ribeiro M.P., Lazzari M., Coutinho P., Otero A. (2021). Biochemical characterization of Nostoc sp. exopolysaccharides and evaluation of potential use in wound healing. Carbohydr. Polym..

[55] El-Baz F.K., Salama A.A.A., Hussein R.A. (2020). Dunaliella salina microalgae oppose thioacetamide-induced hepatic fibrosis in rats. Toxicol. Rep..

[56] Zamani N., Fazilati M., Salavati H., Izadi M., Koohi-Dehkordi M. (2020). The topical cream produced from phycocyanin of Spirulina platensis accelerates wound healing in mice infected with Candida albicans. Appl. Biochem. Microbiol..

[57] Foo S.C., Lee Z.S., Yap M.K.K., Tan J.W. (2023). The antioxidant, wound healing properties and proteomic analysis of water extracts from the tropical cyanobacteria, Nostoc NIES-2111_MUM004. 3 Biotech..

[58] Gunes S., Tamburaci S., Dalay M.C., Deliloglu Gurhan I. (2017). In vitro evaluation of Spirulina platensis extract incorporated skin cream with its wound healing and antioxidant activities. Pharm. Biol..

[59] Hu H., Zhong D., Li W., Lin X., He J., Sun Y., Zhou M. (2022). Microalgae-based bioactive hydrogel loaded with quorum sensing inhibitor promotes infected wound healing. Nano Today.

[60] Chen H., Cheng Y., Tian J., Yang P., Zhang X., Chen Y., Wu J. (2020). Dissolved oxygen from microalgae-gel patch promotes chronic wound healing in diabetes. Sci. Adv..

[61] Jin N., Wu J., Ye S., Xue J., Meng T., Hu L., Zhang G. (2024). Injectable dynamic ROS-responsive COF-modified microalgae gels for in vivo bFGF delivery to treat diabetic wounds. ACS Appl. Mater. Interfaces.

[62] Wu Y., Li M., He R., Xiao L., Liu S., Chen K., Li Y. (2024). Photosynthetic live microorganism-incorporated hydrogels promote diabetic wound healing via self-powering and oxygen production. Chem. Eng. J..

[63] Kang Y., Xu L., Dong J., Yuan X., Ye J., Fan Y., Ji X. (2024). Programmed microalgae-gel promotes chronic wound healing in diabetes. Nat. Commun..

[64] Wu H., Yang P., Li A., Jin X., Zhang Z., Lv H. (2023). Chlorella sp.-ameliorated undesirable microenvironment promotes diabetic wound healing. Acta Pharm. Sin. B.

[65] Chen H., Guo Y., Zhang Z., Mao W., Shen C., Xiong W., Wu J. (2022). Symbiotic algae–bacteria dressing for producing hydrogen to accelerate diabetic wound healing. Nano Lett..

[66] Choi H., Kim B., Jeong S.H., Kim T.Y., Kim D.P., Oh Y.K., Hahn S.K. (2023). Microalgae-based biohybrid microrobot for accelerated diabetic wound healing. Small.

[67] Vazquez-Ayala L., Del Ángel-Olarte C., Escobar-García D.M., Rosales-Mendoza S., Solis-Andrade I., Pozos-Guillén A., Palestino G. (2024). Chitosan sponges loaded with metformin and microalgae as dressing for wound healing: a study in diabetic bio-models. Int. J. Biol. Macromol..

[68] Kumar M., Kumar D., Garg Y., Mahmood S., Chopra S., Bhatia A. (2023). Marine-derived polysaccharides and their therapeutic potential in wound healing application - a review. Int. J. Biol. Macromol..

[69] Hussein R.A., Salama A.A.A., El Naggar M.E., Ali G.H. (2019). Medicinal impact of microalgae collected from high rate algal ponds; phytochemical and pharmacological studies of microalgae and its application in medicated bandages. Biocatal. Agric. Biotechnol..

[70] Singh S., Kumar M., Kumar D., Kumar S., Chopra S., Bhatia A. (2024). Therapeutic precision: unveiling the potential of 3D printing in drug delivery, tissue engineering, and regenerative medicine. 3D Print. Addit. Manuf..

[71] Wang X., Yang C., Yu Y., Zhao Y. (2022).

[72] Kanwal S., De-Eknamkul W. (2023). A non-functional γ-aminobutyric acid shunt pathway in cyanobacterium synechocystis sp. PCC 6803 enhances δ-aminolevulinic acid accumulation under modified nutrient conditions. Int. J. Mol. Sci..

[73] Kanwal S., Incharoensakdi A. (2019). The role of GAD pathway for regulation of GABA accumulation and C/N balance in Synechocystis sp. PCC6803. J. Appl. Phycol..

[74] Kumar S., Marrero-Berrios I., Kabat M., Berthiaume F. (2019). Recent advances in the use of algal polysaccharides for skin wound healing. Curr. Pharm. Des..

[75] Machmud E., Ruslin M., Waris R., Asse R.A., Qadafi A.M., Achmad H. (2020). Effect of the application of chlorella vulgaris ointment to the number of fibroblast cells as an indicator of wound healing in the soft tissue of pig ears. Pesqui. Bras. em Odontopediatria Clínica Integr..

[76] Zhang X., Zhao X., Hua Z., Xing S., Li J., Fei S., Tan M. (2023). ROS-triggered self-disintegrating and pH-responsive astaxanthin nanoparticles for regulating the intestinal barrier and colitis. Biomaterials.

[77] Fang Q., Guo S., Zhou H., Han R., Wu P., Han C. (2017). Astaxanthin protects against early burn-wound progression in rats by attenuating oxidative stress-induced inflammation and mitochondria-related apoptosis. Sci. Rep..

[78] Meephansan J., Rungjang A., Yingmema W., Deenonpoe R., Ponnikorn S. (2017). Effect of astaxanthin on cutaneous wound healing. Clin. Cosmet. Invest. Dermatol..

[79] Veeruraj A., Liu L., Zheng J., Wu J., Arumugam M. (2019). Evaluation of astaxanthin incorporated collagen film developed from the outer skin waste of squid Doryteuthis singhalensis for wound healing and tissue regenerative applications. Mater. Sci. Eng. C.

[80] Oh H., Lee J.S., Sung D., Lim J.-M., Choi W.I. (2020). Potential antioxidant and wound healing effect of nano-liposol with high loading amount of astaxanthin. Int. J. Nanomed..

[81] Kanwugu O.N., Glukhareva T.V., Danilova I.G., Kovaleva E.G. (2022). Natural antioxidants in diabetes treatment and management: prospects of astaxanthin. Crit. Rev. Food Sci. Nutr..

[82] Aneesh P.A., Ajeeshkumar K.K., Lekshmi R.G.K., Anandan R., Ravishankar C.N., Mathew S. (2022). Bioactivities of astaxanthin from natural sources, augmenting its biomedical potential: a review. Trends Food Sci. Technol..

[83] Agustina S., Aidha N.N., Oktarina E., Kurniati N.F. (2021). Evaluation of antioxidant and wound healing activities of Spirulina sp. Extract, Egyptian Journal of Chemistry.

[84] Hussein R.A., Salama A.A., El Naggar M.E., Ali G.H. (2019). Medicinal impact of microalgae collected from high rate algal ponds; phytochemical and pharmacological studies of microalgae and its application in medicated bandages. Biocatal. Agric. Biotechnol..

[85] Hosikian A., Lim S., Halim R., Danquah M.K. (2010). Chlorophyll extraction from microalgae: a review on the process engineering aspects. Int. J. Chem. Eng..

[86] Andryukov B.G., Besednova N.N., Kuznetsova T.A., Zaporozhets T.S., Ermakova S.P., Zvyagintseva T.N., Smolina T.P. (2020). Sulfated polysaccharides from marine algae as a basis of modern biotechnologies for creating wound dressings: current achievements and future prospects. Biomedicines.

[87] Severo I.A., Dias R.R., do Nascimento T.C., Deprá M.C., Maroneze M.M., Zepka L.Q., Jacob-Lopes E. (2022). Microalgae-derived polysaccharides: potential building blocks for biomedical applications. World J. Microbiol. Biotechnol..

[88] De Jesus Raposo M.F., De Morais A.M.B., De Morais R.M.S.C. (2015). Marine polysaccharides from algae with potential biomedical applications. Mar. Drugs.

[89] Premarathna A.D., Ahmed T.A.E., Rjabovs V., Hammami R., Critchley A.T., Tuvikene R., Hincke M.T. (2024). Immunomodulation by xylan and carrageenan-type polysaccharides from red seaweeds: anti-inflammatory, wound healing, cytoprotective, and anticoagulant activities. Int. J. Biol. Macromol..

[90] Ajayi E.I.O., Oladele J.O., Nkumah A.O. (2023). Application of algae in wound healing. Next‐Generation Algae.

[91] Kuznetsova T.A., Andryukov B.G., Besednova N.N., Zaporozhets T.S., Kalinin A.V. (2020). Marine algae polysaccharides as basis for wound dressings, drug delivery, and tissue engineering: a review. J. Mar. Sci. Eng..

[92] Wulandari P.A.C., Ilmi Z.N., Husen S.A., Winarni D., Alamsjah M.A., Awang K., Pudjiastuti P. (2021). Wound healing and antioxidant evaluations of alginate from sargassum ilicifolium and mangosteen rind combination extracts on diabetic mice model. Appl. Sci..

[93] Lu X., Qin L., Guo M., Geng J., Dong S., Wang K., Liu M. (2022). A novel alginate from Sargassum seaweed promotes diabetic wound healing by regulating oxidative stress and angiogenesis. Carbohydr. Polym..

[94] Ilmi Z.N., Wulandari P.A.C., Husen S.A., Winarni D., Alamsjah M.A., Awang K., Pudjiastuti P. (2020). Characterization of alginate from sargassum duplicatum and the antioxidant effect of alginate–okra fruit extracts combination for wound healing on diabetic mice. Appl. Sci..

[95] Zhu F., Du B., Xu B. (2016). A critical review on production and industrial applications of beta-glucans. Food Hydrocoll..

[96] Barsanti L., Gualtieri P. (2023). Glucans, paramylon and other algae bioactive molecules. Int. J. Mol. Sci..

[97] Korolenko T.A., Bgatova N.P., Ovsyukova M.V., Shintyapina A., Vetvicka V. (2020). Hypolipidemic effects of β-glucans, mannans, and fucoidans: mechanism of action and their prospects for clinical application. Molecules.

[98] Yasuda K., Ogushi M., Nakashima A., Nakano Y., Suzuki K. (2018). Accelerated wound healing on the skin using a film dressing with β-glucan paramylon. In Vivo.

[99] Kandhwal M., Behl T., Singh S., Sharma N., Arora S., Bhatia S., Bungau S. (2022). Role of matrix metalloproteinase in wound healing. Am J Transl Res.

[100] Lupette J., Benning C. (2020). Human health benefits of very-long-chain polyunsaturated fatty acids from microalgae. Biochimie.

[101] Gonzaga do Nascimento-Neto L., Carneiro R.F., Da Silva S.R., Da Silva B.R., Arruda F.V.S., Carneiro V.A., Nagano C.S. (2012). Characterization of isoforms of the lectin isolated from the red algae bryothamnion seaforthii and its pro-healing effect. Mar. Drugs.

[102] Lal D.K., Kumar B., Raghav S.S., Bhargava S., Singhal M., Sethiya N.K. (2023). Lectin: a carbohydrate binding glyoprotein and its potential in wound healing. Bioactive Carbohydrates and Dietary Fibre.

